# A new approach for detecting adventitious viruses shows Sf-rhabdovirus-negative Sf-RVN cells are suitable for safe biologicals production

**DOI:** 10.1186/s12896-017-0412-z

**Published:** 2018-02-07

**Authors:** Christoph Geisler

**Affiliations:** GlycoBac LLC, 1938 Harney Street, Laramie, WY 82072 USA

**Keywords:** Adventitious virus, Errantivirus, Endogenous viral element, Maverick/Polinton/Polintovirus, *Spodoptera frugiperda* Sf-RVN, Massively parallel sequencing

## Abstract

**Background:**

Adventitious viral contamination in cell substrates used for biologicals production is a major safety concern. A powerful new approach that can be used to identify adventitious viruses is a combination of bioinformatics tools with massively parallel sequencing technology. Typically, this involves mapping or BLASTN searching individual reads against viral nucleotide databases. Although extremely sensitive for known viruses, this approach can easily miss viruses that are too dissimilar to viruses in the database. Moreover, it is computationally intensive and requires reference cell genome databases. To avoid these drawbacks, we set out to develop an alternative approach. We reasoned that searching genome and transcriptome assemblies for adventitious viral contaminants using TBLASTN with a compact viral protein database covering extant viral diversity as the query could be fast and sensitive without a requirement for high performance computing hardware.

**Results:**

We tested our approach on *Spodoptera frugiperda* Sf-RVN, a recently isolated insect cell line, to determine if it was contaminated with one or more adventitious viruses. We used Illumina reads to assemble the Sf-RVN genome and transcriptome and searched them for adventitious viral contaminants using TBLASTN with our viral protein database. We found no evidence of viral contamination, which was substantiated by the fact that our searches otherwise identified diverse sequences encoding virus-like proteins. These sequences included Maverick, R1 LINE, and errantivirus transposons, all of which are common in insect genomes. We also identified previously described as well as novel endogenous viral elements similar to ORFs encoded by diverse insect viruses.

**Conclusions:**

Our results demonstrate TBLASTN searching massively parallel sequencing (MPS) assemblies with a compact, manually curated viral protein database is more sensitive for adventitious virus detection than BLASTN, as we identified various sequences that encoded virus-like proteins, but had no similarity to viral sequences at the nucleotide level. Moreover, searches were fast without requiring high performance computing hardware. Our study also documents the enhanced biosafety profile of Sf-RVN as compared to other Sf cell lines, and supports the notion that Sf-RVN is highly suitable for the production of safe biologicals.

**Electronic supplementary material:**

The online version of this article (doi: 10.1186/s12896-017-0412-z) contains supplementary material, which is available to authorized users.

## Background

Adventitious viruses have been found to contaminate cell substrates used in biologicals production on several occasions, and are considered a major safety concern [1]. In response, a variety of methods have been developed to probe for viruses in cell substrates and other materials used in biologicals production [2, 3]. One approach that can be used to probe for adventitious viruses is massively parallel sequencing (MPS) combined with read mapping or BLASTN searches against viral nucleotide sequence databases [4–8]. The lack of sequence bias and depth of sequence coverage provide compelling arguments for the use of MPS in this application.

Although this approach is highly suited for the detection of known viruses, it can easily miss viruses that are too dissimilar to viruses in the search database. Another drawback is the requirement for high performance computing hardware, as it is computationally intensive. Furthermore, to be effective, host cell reads need to be filtered from the MPS data prior to further analysis, leading to a requirement for high quality reference genome databases [4, 9, 10]. Such databases are only available for a few select species.

To avoid these drawbacks, we set out to develop an alternative approach to search MPS data for adventitious viral sequences. We reasoned that TBLASTN searching genome and transcriptome assemblies, not individual reads, against a compact custom database comprising a comprehensive set of viral proteins from an inclusive range of viruses (viral protein database, VPD) could be sensitive and computationally relatively non-intensive without a requirement for high quality reference genome databases. This workflow is outlined in Fig. 1.

**Fig. 1:** Workflow of the approach presented in this paper

We tested our approach on Sf-RVN, a recently isolated *Spodoptera frugiperda* (Sf) insect cell line [11]. Unlike other Sf cell lines, Sf-RVN is not persistently infected with Sf-rhabdovirus [12–14]. Sf-RVN cells lack phenotypes commonly associated with viral infection, such as nuclear hypertrophy, inclusion bodies, or syncytia formation. However, insect cell lines known to be persistently infected with adventitious viruses also lack these phenotypes. Moreover, insects and insect cell lines can be simultaneously infected with multiple viruses [15, 16]. Thus, we wanted to test the possibility that Sf-RVN cells are persistently infected with adventitious viruses other than Sf-rhabdovirus.

We assembled the Sf-RVN cell genome and transcriptome using Illumina MPS reads, and searched the resulting contigs for sequences encoding virus-like proteins using TBLASTN with our VPD as the query. Both the genome and transcriptome were queried to identify potential latent DNA virus infections, and to correctly classify transcribed endogenous viral elements (EVEs) and other transcribed virus-like genomic sequences [17]. Finally, we searched the Sf-RVN genome and transcriptome for errantiviruses using previously published Sf cell and lepidopteran errantivirus sequences as the query.

Our BLAST searches did not reveal evidence of contamination with Sf-rhabdovirus or any other viruses. However, they did identify diverse sequences encoding virus-like proteins. These included Maverick and R1 LINE DNA transposons, as well as several previously partially described [18] errantiviral sequences. Our TBLASTN searches also identified previously described Sf-rhabdovirus-like EVEs [17], as well as several new EVEs similar to ORFs encoded by diverse insect viruses.

We conclude that our approach to probe MPS assemblies for adventitious viruses using TBLASTN with a manually curated, compact viral protein database is not only fast, but also highly sensitive, as we identified various sequences that encoded virus-like proteins, but had no similarity to viral sequences at the nucleotide level. Furthermore, considering these searches identified diverse virus-like sequences, but no sequences associated with typical replication-competent viruses, we conclude Sf-RVN is not contaminated with Sf-rhabdovirus or any other viral adventitious agents.

## Methods

### Cell culture, DNA and RNA extraction, MPS

Sf-RVN cells (GlycoBac, Laramie, WY, USA) were routinely maintained as previously described [11]. DNA and RNA were extracted as previously described [17]. DNA and RNA library preparations, sequencing reactions, and initial bioinformatics analysis were conducted by Genewiz, LLC (South Plainfield, NJ, USA), as described below.

For transcriptome sequencing, an RNA library was prepared using the NEBNext Ultra RNA Library Prep Kit for Illumina (E7530, New England Biolabs) following the manufacturer’s recommendations. PolyA+ mRNAs were enriched from total RNA with oligo d (T) beads, as kits that selectively degrade rRNA using species-specific rRNA-complementary DNA probes with RNAseH are not available for, or are untested with lepidopteran insect RNA samples. It is conceivable RNAs from the few viruses that do not produce polyadenylated RNAs were depleted during the polyA+ enrichment step, and that such viruses, if present, could consequently escape detection. Given the circumstances, we felt rRNA depletion through polyA+ enrichment was a necessary compromise. However, it should be noted recent research indicates several viruses previously thought not to produce polyadenylated RNAs do in fact produce polyA+ RNA at a low frequency [19, 20], suggesting that RNA from such viruses may still be detected.

Following polyA+ enrichment, RNAs were fragmented for 15 min at 94 °C. First and second strand cDNA’s were subsequently synthesized, cDNA fragments were end repaired and 3′-adenylated, and universal adapters were ligated to cDNA fragments. For genome sequencing, a DNA library was prepared using the NEBNext Ultra DNA Library Prep Kit for Illumina (E7370, New England Biolabs) following the manufacturer’s recommendations. Briefly, the genomic DNA was fragmented by acoustic shearing with a Covaris S220 ultrasonicator, end repaired and 3′-adenylated, and universal adapters were ligated to DNA fragments.

Adapter-ligated DNAs were indexed and enriched by limited cycle PCR, quantified by real-time PCR, and multiplexed by equal molar mass. Pooled libraries were clustered onto a flowcell lane and loaded on the Illumina HiSeq 2500 instrument according to the manufacturer’s instructions, and were sequenced using a 2 × 150 paired-end (PE) Rapid Run configuration. Image analysis and base calling were conducted by the HiSeq Control Software (HCS) on the HiSeq2500 instrument and raw sequence data was converted into the fastq format and de-multiplexed using the Illumina CASAVA 1.8.2 program. One mismatch was allowed for index sequence identification. FastQ files from each sample were trimmed to remove adapter sequences and poor quality reads at the ends. De novo assembly was conducted using CLC Genomics Server 8.0.3 and the resulting reads were assembled in CLC Genomics Workbench. Finally, the resulting assemblies were uploaded to GenBank (BioProject PRJNA344686).

### BLAST searches

Searchable Sf-RVN genome and transcriptome databases were generated using the NCBI BLAST+ suite, and queried through the prfectBLAST Java front end [21] (BLAST+ version 2.4.0) with an in-house viral protein database (see below) through TBLASTN searches. Search results with an E-value <0.1 were further investigated by comparing translated sequences to the NCBI Conserved Domain Database (CDD) [22] to identify domains that could aid in classifying sequences as viral or insect. Search results were also classified by comparing contigs to viral and insect proteins in the GenBank database through BLASTX searches. If insect proteins were much more similar than the most closely related viral proteins, contigs were classified as insect, not viral sequences. Typically, if a predicted protein was a conserved insect protein, proteins from related insect species had E values tens of orders of magnitude lower than viral proteins.

### Sequence comparison

Amino acid alignments were automatically generated using ClustalX2 [23] and manually corrected, as required. Protdist (PHYLIP Version 3.695) was used to generate distance matrices with the Jones-Taylor-Thornton model. Unrooted trees were then generated using the neighbor-joining method (Neighbor; PHYLIP package) and drawn using the PHYLIP drawtree postscript generator.

## Results

### Sf-RVN cell genome and transcriptome assembly

The assembled Sf-RVN cell genome comprised 392 Mb in 66,319 contigs at approximately 121-fold coverage, and the assembled Sf-RVN cell transcriptome comprised 39.6 Mb in 22,370 contigs at 548-fold coverage (for additional details, see Table 1). These numbers are comparable to those associated with the previously released draft genome and transcriptome of *S. frugiperda* Sf21 cells, which comprised 358 Mb in 37,235 contigs, and 47.4 Mb in 24,016 contigs, respectively [24, 25]. However, our genome assembly had only 0.55% of N’s in gaps, whereas the previously released draft had 7.7% of N’s in gaps. Thus, our genome assembly has fewer and shorter gaps, although our N50 (12.4 kB) is shorter than the N50 of the previously released draft genome (53.7 kB). This latter disparity can be at least partially attributed to the use of three datasets for the previously released draft genome [24]. These included a short insert (350 bp) paired end (100 bp) library (Illumina), a single read (average read length of 300 bp) library (Roche Titanium), and a long insert (2 kbp) paired end (60 bp) library (ABI SOLiD). The use of these three libraries allowed Kakumani et al. [24] to assemble larger supercontigs than we could using only a single 150 bp paired end library. For our transcriptome, the N50 (2.6 kb) was also somewhat shorter than that of the recently published Sf21 cell transcriptome (3.4 kb). Overall, the quality of our assembled genome and transcriptome is comparable to the previously released Sf21 cell draft genome and transcriptome.

**Table 1:** Sf-RVN MPS results summary

	Genome	Transcriptome
Yield (Gb)	50.8	46.7
Reads × 10^6^	493.4	453.4
Coverage (fold)	120	548
% of Q Scores ≥Q30	92.8	94.6
Mean Q score	37.7	38.2
Contigs/scaffolds	66,319	22,370
Maximum length (bps)	202,654	21,539
Minimum length (bps)	490	436
N50 (bps)	12,380	2576
Average contig length (bps)	5906	1770
Total bases in assembly (Mbps)	391.6	39.6
Total base reads × 10^9^	48.7	24.5
Matched base reads × 10^9^	47.2	21.7

### Viral protein database (VPD) construction

As protein sequences are far more highly conserved than nucleotide sequences, we searched the Sf-RVN cell genome and transcriptome using TBLASTN searches [26] with a custom viral protein database (VPD) as the query. At the time of this writing, the NCBI GenBank database contained approximately 4.2 million viral protein sequences, as determined by using (viruses [filter]) as the search term. Using a VPD containing all these sequences as the query for TBLASTN searches would be computationally very intensive. The redundancy introduced by variants with only minor differences, duplicates and incomplete sequences would also complicate interpretation of the search results.

Thus, we created an in-house VPD containing viral proteins from at least one representative of all virus families in the Baltimore classification, as described in the Virus Taxonomy: 2015 Release by the International Committee on Taxonomy of Viruses (http://www.ictvonline.org/virustaxonomy.asp), as well as proteins from at least one virus for each unclassified virus family. We used ‘type’ viruses if their whole genome had been sequenced. Otherwise, we used another virus whose whole genome had been sequenced to represent that family. We also included viruses known to be able to infect *S. frugiperda*, such as Sf-rhabdovirus, as well as viruses known to contaminate insect cell cultures, such as *Bombyx mori* macula-like latent virus [27–30].

Finally, we manually curated our VPD to account for the fact that viral proteins often have sequences similar to host cell proteins. For example, a comparison of the *B. mori* nuclear polyhedrosis virus (BmNPV) and *B. mori* proteomes showed 15 of 136 BmNPV proteins (11%) have significant similarity to *B. mori* proteins [31], with BLASTP E values as low as 2e-79. Thus, we removed all viral protein sequences with close eukaryotic cellular homologs. Most were proteins or protein subunits containing conserved domains found in DNA and RNA polymerases, kinases, phosphatases, apoptosis inhibitors, superoxide dismutases, proteases, nucleases, ubiquitin ligases, DNA binding proteins (zinc or ring fingers), and others. The resulting curated VPD contained 6981 protein sequences from 363 different viruses.

Next, we used the VPD as the query in TBLASTN searches against the assembled contigs in the Sf-RVN cell genome and transcriptome, as described. Our TBLASTN searches revealed that there was no homology between a majority of proteins in the VPD and proteins putatively encoded by assembled Sf-RVN sequences. However, our TBLASTN searches also determined that several Sf-RVN sequences encoded putative proteins with significant homology to proteins in the VPD.

Based on further bioinformatics analysis, we determined that these Sf-RVN sequences comprised Maverick/Polinton elements, R1 LINEs, or endogenous viral elements (EVEs). In the following sections, we describe the TBLASTN search results that revealed Sf-RVN sequences encoding putative proteins with significant similarity to specific viral proteins, and how we determined they do not constitute (parts of) replication competent viruses.

### Maverick / Polinton elements

Maverick transposable elements [32, 33], also known as Polintons [34], are a novel class of giant transposable elements that are distantly related to various DNA viruses. Although absent from mammals [33], Maverick elements are widespread in eukaryotes and have been identified previously in various insect orders including Lepidoptera [35].

Surprisingly, we were able to identify Mavericks in Sf-RVN cells through their distant similarity to viral sequences included in our VPD. TBLASTN searching the Sf-RVN cell genome and transcriptome using our VPD revealed contigs with highly significant similarity (E values 4e-67 and higher) to proteins from *C. congregata* bracovirus, *M. sanguinipes* entomopoxvirus, *B. mori* densovirus, and other dsDNA viruses. These contigs could be assembled into supercontigs containing at least nine putative ORFs (Fig. 2, See Additional file 1, Sf-Mavericks; Genbank accession numbers KY042018 and KY042019). The predicted products of five of these ORFs were assigned putative functions based on annotations by the NCBI Conserved Domain Database (CDD) [22]. Conforming to established nomenclature [34], these were: (1) ATP, which was similar to the poxvirus A32 ATPase; (2) INT, which was similar to retroviral integrase, (3) PRO, which was similar to adenoviral cysteine protease, (4) POLB, which was similar to DNA polymerase B2, and (5) CAP, which was similar to parvovirus VP1 (Fig. 2). The presence of five ORFs with these putative functions is a hallmark of a type of DNA transposon referred to as Polintons [34] or Mavericks [32, 33], which typically comprise a total of six to ten ORFs [33].

**Fig. 2:** Structure and relative sizes of Sf Maverick 1 and 2 elements. ORFs conserved among Sf Maverick 1 and 2 are indicated: ORFs encoding putative proteins with conserved domains are shaded in light gray (ATP, INT, CAP, PRO and POLB), and ORFs that do not contain identifiable domains are shaded in dark gray (ORF2, ORF6-8)

Because the assembled supercontigs included a number of putative ORFs that is typical for Mavericks, because they contained the five canonical Maverick ORFs, and because they were similar in size and organization to previously described Mavericks, we tentatively concluded Sf-RVN cells contain Maverick elements.

The presence of two distinct Maverick lineages in a single genome was previously reported to be a common occurrence [34, 36]. In the present study, we also identified two distinct lineages of apparently intact Maverick elements: one with a series of 8 small tandem ORF’s and a larger ORF encoded by the same DNA strand (‘Sf Maverick 1’), and a second with a similar series of 8 small tandem ORFs, followed by a larger ORF encoded by the opposite strand (‘Sf Maverick 2’) (Fig. 2). The 8 smaller tandem ORFs had the same order in the two lineages. The 9 ORFs encoded by the two Maverick lineages were related, but clearly distinct, and the predicted amino acid sequences were only 52% identical on average (Table 2). We also identified other partial Maverick sequences closely related to Sf-RVN Maverick 1 or 2 in genomic and transcriptomic contigs, but could not determine if these were part of intact Maverick elements.

**Table 2:** Similarity among Sf-Maverick 1 and 2 ORFs

	Amino acid identity	Amino acid similarity	BLASTP amino acids aligned	BLASTP E value	BLASTN nucleotides aligned	BLASTN E value
POLB	52%	72%	All / 1162	0	1916 / 3498	1e-102
ATP	59%	79%	All / 228	8e-107	471 / 684	3e-49
ORF2	37%	58%	All / 305	4e-63	119 / 918	1e-20
INT	60%	75%	All / 310	2e-133	748 / 930	2e-56
CAP	55%	69%	250 / 258	3e-90	396 / 774	2e-28
PRO	57%	71%	120 / 133	1e-51	365 / 408	3e-13
ORF6	30%	40%	134 / 148	2e-31	–	–
ORF7	59%	77%	391 / 404	0	459 / 1215	1e-28
ORF8	44%	66%	149 / 158	8e-49	–	–

We initially noticed the predicted translation products of several Sf-RVN contigs were highly similar to proteins encoded by *C. congregata* bracovirus (*Polydnaviridae*), which at first led us to believe Sf-RVN cells contained polydnaviral DNA. However, after more detailed analysis, we realized this similarity was caused by the presence of a partial Maverick element in a *C. congregata* bracovirus proviral circle [35] that was similar to the Sf-RVN Mavericks. Thus, we concluded Sf-RVN cells are not persistently infected with a bracovirus.

#### B2 DNA polymerase (POLB)

Like previously described Mavericks, Sf Maverick 1 and 2 contain large ORFs (~3500 bps) that appear to encode proteins with B2 DNA polymerase (POLB) domains between amino acid residues 500–1000, based on annotation by the NCBI CDD (Table 3). Remarkably, TBLASTN searches revealed Sf Maverick POLBs were very similar to *Bombyx mori* densovirus DNA polymerase (Table 4). However, this similarity did not extend beyond the ~500 amino acids of the DNA polymerase B2 domains, and the N-terminal halves of the Sf Maverick POLBs and densovirus DNA polymerase had no similarity. Finally, we found Sf Maverick POLBs were also weakly similar to various mammalian adenovirus DNA polymerases (Table 4).

**Table 3:** Sf-Maverick 1 and 2 ORF domains as annotated by comparison to the CDD

ORF	Domain	Sf Maverick 1 E value	Sf Maverick 2 E value
ATP	AAA ATPase domain	9.76e-04	2.3
	Poxvirus A32-like	0.03	–
INT	Integrase core domain	4.22e-12	5.86e-16
	Chromo domain	6.01e-04	3.45e-04
CAP	Parvovirus coat protein VP1	4.23e-04	8.15e-04
	Phospholipase A2 (PLA2)	3.52e-04	0.04
PRO	Adenovirus endoprotease	6.1	0.58
	Serine protease	0.51	–
POLB	DNA polymerase B2	2.08e-14	5.92e-17
	Recombination endonuclease VII	0.02	0.32

**Table 4:** Sf Maverick 1 and 2 ORF protein similarity to GenBank viral proteins: lowest E values are listed

ORF	Viruses	Sf Maverick 1 E value	Sf Maverick 2 E value
ATP	Mammalian poxviruses	2e-05	3e-04
	Entomopoxviruses	8e-04	2e-04
INT	Mammalian retroviruses	5e-05	1e-09
CAP	Entomopoxviruses	3e-10	1e-10
	Mammalian parvoviruses	4e-04	5e-06
	Insect densoviruses	2e-05	3e-06
PRO	Mammalian adenoviruses	4e-04	6e-05
POLB	*Bombyx mori* densovirus	6e-58	4e-67
	Mammalian adenoviruses	0.13	0.004

Figure 3a shows an amino acid alignment of the Sf Maverick 1 and 2 POLB proteins and the *B. mori* densovirus 3 DNA polymerase, with domains based on annotations by the NCBI Conserved Domain Database (CDD) indicated. Figure 3b shows the results of a phylogenetic analysis demonstrating the relationship among Sf Maverick POLB proteins, other insect and previously identified vertebrate Maverick POLBs [34], and *B. mori* densovirus POLB. Sf Maverick 1 and 2 POLB clustered closely with other insect Maverick POLBs, whereas vertebrate Maverick and *B. mori* densovirus POLBs formed distinct outgroups. Thus, Sf Maverick 1 and 2 POLB are much more closely related to other insect Maverick POLBs than to *B. mori* densovirus POLB, which among viral proteins is by far the most similar to Sf Maverick POLBs (Table 4). The close clustering of Sf Maverick 1 and 2 POLB with other putative insect Maverick POLB proteins supports the conclusion that Sf Maverick POLBs, though relatively closely related to *B. mori* densovirus POLB, are not densoviral sequences, but components of insect Maverick elements.

**Fig. 3:** Sf-RVN cell Maverick 1 and 2 POLB are more similar to homologous proteins encoded by other Mavericks than to related viral proteins. **a** Amino acid alignment of the Sf Maverick 1 and 2 POLB proteins and the *B. mori* densovirus 3 DNA polymerase. The predicted Recombination Endonuclease VII and DNA POLB2 domains are indicated. **b** Unrooted tree showing the phylogenetic relationships among Sf Maverick and other insect and vertebrate Maverick POLB proteins, and *B. mori* densovirus 3 DNA polymerase. Abbreviations: At, the navel orangeworm *Amyelois transistella*; Bm, the silkworm *Bombyx mori*; Dr, the zebrafish *Danio rerio*; Px, the diamondback moth *Plutella xylostella*; Sc, the stable fly *Stomoxys calcitrans*; Sf, the fall armyworm *Spodoptera frugiperda* (this study); Tc, the flour beetle *Tribolium castaneum*

#### ATPase (ATP)

Comparison to the NCBI CDD revealed Sf Mavericks, like previously described Maverick elements, contain ORFs encoding putative proteins similar to AAA+ ATPases (ATP, Table 3). BLAST searches against viral proteins showed Sf Maverick 1 and 2 ATP were most similar to mammalian poxvirus A32-like proteins (Table 4), which are ATPases involved in packaging DNA into viral particles [37, 38]. Predicted entomopox virus ATPase proteins also had weak similarity to Sf-Maverick ATPs (Table 4). Figure 4a shows an amino acid alignment of Sf Maverick 1 and 2 ATPs with a zebrafish Maverick ATP, cowpox virus A32 ATP, and *A. honmai* entomopoxvirus ATP. Amino acids demonstrated to be involved in ATP binding and coordination (Walker A and B motifs) [39, 40] are fully conserved among these sequences, suggesting Sf Maverick 1 and 2 ATP are bona fide ATPases.

**Fig. 4:** Sf-RVN cell Maverick 1 and 2 ATP and CAP are more similar to homologous proteins encoded by other Mavericks than to related viral proteins. **a** Amino acid alignment of the AAA+ ATPase domain regions of Sf Maverick 1 and 2 ATP, vertebrate Maverick ATP, cowpox virus A32 ATPase, and *A. honmai* entomopoxvirus ATPase. Conserved amino acid residues that constitute the ATPase Walker A and B motifs are indicated with a filled circle. **b** Unrooted tree showing the phylogenetic relationships among Sf Maverick and other insect and vertebrate Maverick ATP proteins, cowpox virus A32 ATPAse and *A. honmai* entomopoxvirus ATPase. **c** Amino acid alignment of the N-terminal regions containing the PLA2 domain of Sf Maverick 1 and 2 CAP, human parvovirus B19 capsid, *B. mori* densovirus 1 capsid, and *A. honmai* entomopoxvirus capsid-like protein. Conserved amino acids involved in catalysis are indicated with a filled circle, those involved in Ca2+ cofactor binding with an asterisk, and those that are otherwise conserved with an plus sign. **d** Unrooted tree showing the phylogenetic relationships among Sf Maverick and other insect Maverick CAP proteins, human parvovirus B19 capsid, *B. mori* densovirus 1 capsid, and *A. honmai* entomopoxvirus capsid-like protein. Abbreviations: Ah, the summer fruit tortix *Adoxophyes honmai*; At, the navel orangeworm *Amyelois transistella*; Bm, the silkworm *Bombyx mori*; Dr, the zebrafish Danio rerio; Ln, the black garden ant *Lasius niger*; Px, the diamondback moth *Plutella xylostella*; Sf, the fall armyworm *Spodoptera frugiperda* (this study); Tc, the flour beetle *Tribolium castaneum*

Figure 4b shows the results of a phylogenetic analysis demonstrating the relationship among Sf Maverick ATP proteins, other insect and previously identified vertebrate Maverick ATP proteins [34], and viral ATP proteins. Sf Maverick 1 and 2 ATPs clustered closely with other insect Maverick ATPs. A second cluster contained the vertebrate Maverick ATPs, as well as two other insect Maverick ATPs. The viral ATP proteins formed a distinct outgroup, indicating Sf Maverick 1 and 2 ATP are more closely related to other insect Maverick ATPs than to poxvirus ATPs, which among viral proteins are the most similar to Sf Maverick ATPs (Table 4). The close clustering of Sf Maverick 1 and 2 ATP with other putative insect Maverick ATPs supports the conclusion that Sf Maverick ATPs, though related to entomopox and other viral ATPases, are components of insect Maverick elements.

#### Capsid-like (CAP)

Surprisingly, Sf Mavericks do not encode a protein homologous to the Maverick PY protein, which is conserved among previously described Maverick elements [34] and has been suggested to contain the double jelly-roll fold found in the capsid proteins of some viruses [41]. Instead, Sf Mavericks encode a different viral capsid-like protein. Comparison to the NCBI CDD revealed the N-terminal region of the putative protein encoded by the 4th small ORF of Sf Maverick 1 and 2 was similar to parvovirus VP1 capsid proteins (Table 3). Thus, we called this protein CAP to distinguish it from previously described Maverick PY ORFs, which also encode capsid-like proteins.

Both invertebrate [42, 43] and vertebrate [44] parvovirus VP1 capsid proteins encode proteins with phospholipase A2 (PLA2) domains, which were also present in the the N-terminal regions of Sf Maverick 1 and 2 CAPs (PLA2, Table 3).

BLAST searches against viral proteins revealed capsid-like proteins from various entomopoxviruses had the highest level of similarity to Sf Maverick 1 and 2 CAP, with the *Adoxophyes honmai* NPV [45] capsid-like protein scoring highest (Table 4). Finally, we found Sf Maverick CAPs were also weakly similar to insect densovirus and mammalian parvovirus capsid proteins (Table 4), which both have PLA2 activity [42–44, 46].

Figure 4c shows an alignment of Sf Maverick CAP proteins, *A. honmai* NPV capsid-like protein, *B. mori* densovirus 1 capsid protein, and human parvovirus B19 VP1 [47, 48]. Residues of the PLA2-like region associated with catalysis and cofactor binding [44, 46] are conserved among Sf Maverick 1 and 2 CAP and the viral capsid proteins, suggesting Sf Maverick 1 and 2 CAP are bona fide phospholipases. The results of a phylogenetic analysis of the relationships among Sf Maverick 1 and 2 CAP, various insect Maverick CAP proteins, *B. mori* densovirus 1, *A. honmai* NPV, and human parvovirus B19 capsid are shown in Fig. 4d. Insect Maverick CAPs cluster closely together, supporting the conclusion that Sf Maverick CAPs, though related to various insect virus capsid proteins, are in fact components of insect Maverick elements.

#### Integrase (INT)

Like other Mavericks, Sf Mavericks contain ORFs encoding putative proteins with an integrase (INT) core-like domain, based on annotation by the NCBI CDD (Table 3). An amino acid alignment of Sf Maverick 1 and 2 INT with a zebrafish Maverick INT and the HIV integrase core domain, for which the catalytic amino acid residues have been mapped [49], is shown in Fig. 5a. These catalytic amino are conserved in retroviruses and class I and II transposon integrases [49, 50]. Figure 5a shows these amino acid residues are also conserved in Sf Maverick 1 and 2 INT, suggesting they are bona fide integrases. Both Sf Maverick 1 and 2 INT also contained a putative chromo domain on their C-termini (Table 3), which is not present in the zebrafish or other previously described Maverick INT proteins. Integrase chromo domains are commonly fused to transposon integrases and have been shown to mediate protein-nucleic acid interactions [51], target site selection [52, 53], and transposition activity [53–55]. Thus, although chromo domains have not previously been reported in Maverick integrases, our finding is not unexpected.

**Fig. 5:** Sf-RVN cell Maverick 1 and 2 INT and PRO are more similar to homologous proteins encoded by other Mavericks than to related viral proteins. **a** Amino acid alignment of the conserved integrase domain containing regions of Sf Maverick 1 and 2 INT, vertebrate Maverick CAP, and HIV integrase. Conserved amino acids involved in catalysis are indicated with a filled circle. **b** Unrooted tree showing the phylogenetic relationships among Sf Maverick and other insect and vertebrate Maverick INT proteins, and HIV integrase. **c** Amino acid alignment of the conserved cysteine endoprotease domain contraining regions of Sf Maverick 1 and 2 PRO, vertebrate Maverick PRO, and adenovirus adenain. Conserved amino acids involved in catalysis are indicated with a filled circle. **d** Unrooted tree showing the phylogenetic relationships among Sf Maverick and other insect and vertebrate Maverick PRO proteins, and adenovirus adenain. Abbreviations: At, the navel orangeworm *Amyelois transistella*; Bm, the silkworm *Bombyx mori*; Dr, the zebrafish *Danio rerio*; Ln, the black garden ant *Lasius niger*; Px, the diamondback moth *Plutella xylostella*; Sc, the stable fly *Stomoxys calcitrans*; Sf, the fall armyworm *Spodoptera frugiperda* (this study); Tc, the flour beetle *Tribolium castaneum*

The results of a phylogenetic analysis of the relationships among Sf Maverick 1 and 2 INT, various insect and vertebrate Maverick, and HIV INT are shown in Fig. 5b. Sf Maverick 1 and 2 INT clustered closely with the other Maverick INTs and a viral INT formed a distinct outgroup. This indicates Sf Maverick 1 and 2 INT are much more closely related to other Maverick INTs than to viral INT (Table 4), and supports the conclusion that Sf Maverick INTs, though related to retroviral integrases, are components of insect Maverick elements.

#### Protease (PRO)

Like previously described Maverick elements, Sf Mavericks also contain ORFs encoding predicted proteins with an adenovirus cysteine endoprotease-like (PRO) domain (Table 3). An alignment of Sf Maverick 1 and 2 PRO with a zebrafish Maverick PRO and the endoprotease domain from adenovirus adenain is shown in Fig. 5c. This alignment demonstrates amino acids forming the catalytic triad in adenain [56] are fully conserved among these sequences, suggesting Sf Maverick 1 and 2 PRO are indeed bona fide proteases.

The results of a phylogenetic analysis of the relationships among Sf Maverick 1 and 2 PRO, various insect and vertebrate Maverick PROs, and adenain are shown in Fig. 5d. Sf Maverick 1 and 2 PRO clustered closely with other insect Maverick PROs, and the vertebrate Maverick PROs and adenovirus adenain formed two distinct outgroups. This indicates Sf Maverick 1 and 2 PRO are more closely related to other insect Maverick PROs than to adenovirus proteases, which among viral proteins are the most similar to Sf Maverick PROs (Table 4). The close clustering of Sf Maverick 1 and 2 PRO with other putative insect Maverick PROs supports the conclusion that Sf Maverick PROs, though related to adenoviral capsid maturation proteases, are components of insect Maverick elements.

### R1 LINEs with virus-like C-terminal superfamily 1 helicase (S1H) domains

Long interspersed nuclear elements (LINEs) are non-long terminal repeat (LTR) transposable elements that are ubiquitous in the genome of many eukaryotes, including lepidopteran insects [57, 58].

TBLASTN searching the Sf-RVN cell genome and transcriptome using our VPD revealed contigs with highly significant similarity (E values 3e-25 and higher) to proteins from positive-sense single-stranded RNA viruses. Surprisingly, proteins from various (+) ssRNA viruses were similar to the same set of Sf-RVN sequences. Comparison to the NCBI CDD revealed the similarity between these translated Sf-RVN sequences and (+) ssRNA virus proteins was limited to regions predicted to encode superfamily 1 RNA helicase (S1H) domains [59, 60].

Recently, Lazareva et al. described lepidopteran R1 long interspersed nuclear elements (LINEs) that were unusual in that the protein encoded by their second large ORF contained a C-terminal S1H domain [58]. Lazareva et al. already noted the extensive similarity of the lepidopteran R1 LINE S1H domains to plant viruses of the genus Tobamovirus and concluded these LINE’s had likely acquired their SH1H domains from (+) ssRNA viruses.

We assembled a complete Sf-RVN R1 LINE sequence, with an overall size and structure very similar to those of the lepidopteran R1 LINE’s with S1H domains previously described by Lazareva et al. [58] (Fig. 6a, see Additional file 1, Sf-R1 LINEs; Genbank accession number MF327145). Figure 6b shows an alignment of the S1H domains of the Sf R1 LINE ORF2, *P. xylostella* R1 LINE ORF2 [58], and the tobacco mosaic virus (TMV) and Negev virus [61] replicases. The latter two were included because it was previously noted TMV replicase was similar to lepidopteran R1 LINEs [58] and Negev virus replicase was the most similar among viral proteins in the NCBI database to Sf R1 LINE ORF2. Figure 6b demonstrates the extensive similarity among the S1H domains and conservation of the characteristic S1H motifs [59], suggesting lepidopteran R1 LINEs contain bona fide S1H domains.

**Fig. 6:** Sf-RVN cell R1 LINE transposons encode proteins with SF1H domains that are more similar to previously identified insect R1 LINE ORF2 proteins with C-terminal SF1H helicase domains, than to proteins from (+)ssRNA viruses. **a** Domain structure and relative size of full-length Sf-RVN and *Plutella xylostella* R1 LINE with SF1H domain. The size and order of conserved domains in ORF2 are very similar. **b** Predicted amino acid sequence alignment of SF1H domains of Sf-RVN and *Plutella xylostella* R1 LINEs, and Negev virus (YP_009256205.1) and TMV replicase (NP_597746.1). The shading is proportional to the degree of amino acid conservation. **c** Phylogenetic analysis of newly identified Sf-RVN and *Plutella xylostella* R1 LINE SF1H domains, and Negev virus and TMV replicase. The LINEs cluster closely together in a group that is distant from ssRNA viruses

Figure 6c shows the results of a phylogenetic analysis demonstrating the relationship among S1H domains of the TMV and Negev virus replicases, and previously described *P. xylostella* [58] (Px LINE) and Sf-RVN R1 LINE ORF2 proteins identified in this study, including those from LINEs that could not be completely assembled (Sf LINE 1, 2, 5, 6, and 7, see Additional file 1, Sf-R1 LINEs). S1H domains of Sf-RVN R1 LINEs and of the lepidopteran insect *P. xylostella* clustered closely together. In contrast, the (+) ssRNA virus S1H domains formed distant outgroups. These observations further support the conclusion that Sf cell S1H sequences, though related to (+) ssRNA viruses, are components of R1 LINE transposons. Thus, the presence of S1H domains in the SfRVN cell genome and transcriptome does not indicate viral contamination.

### Novel EVEs

Finally, TBLASTN searching the Sf-RVN cell genome and transcriptome using our VPD revealed contigs that were highly similar to proteins from various (−) ssRNA viruses (Table 5, see Additional file 1, Sf-EVEs). Considering (−) ssRNA viruses do not have a DNA stage in their lifecycle, and considering the same sequences could be identified in both the genome and the transcriptome, we classified these sequences as endogenous viral elements (EVEs). We identified five new EVEs in Sf-RVN cells, and also detected the four EVEs previously described in this cell line [17] (Table 5).

**Table 5:** Summary of EVEs in Sf-RVN cells

EVE	Highest BLASTN E value	Highest TBLASTX E value	Length (bps)	Nonsense/rameshift mutations	RPKM	Reads mapped
Maraba virus L-like	6e-39	2e-59	493	1 / 1	0	0
Orinoco virus L-like	4.5 ^a^	3e-42	280	0 / 1	571	105
Taï virus N-like	3.2 ^a^	2e-22	534	0 / 0	29 × 10^3^	13,355
*Pararge aegeria* rhabdovirus N-like	0.69 ^a^	7e-17	540	4 / 0	0	0
Shuangao insect virus 3 G-like	0.67 ^a^	4e-36	1551	0 / 0	5.6	6
Sf-rhabdovirus N-like			1503	0 / 0	4.0	4
Sf-rhabdovirus P-like			1137	0 / 0	19	14
Sf-rhabdovirus G-like			1131	0 / 0	2.8	2
Sf-rhabdovirus L-like			1259	0 / 0	12	10

^a^hits were to irrelevant viral sequences

Two of the newly discovered EVEs encode predicted translation products similar to mononegaviral L proteins (Table 5). The predicted translation product of the first L-like EVE (Genbank accession number MF327146) is most similar to the L protein from Maraba virus, a vesiculovirus isolated from phlebotomine sand flies [62, 63]. This product is also similar to a large number of rhabdoviral L proteins, as it comprised a conserved region of this protein. The predicted translation product of the second L-like EVE (Genbank accession number MF327147) is most similar to the L protein of Orinoco virus, a rhabdovirus isolated from the green pug, which is a moth (*Pasiphila rectangulata*). This product is also similar to L proteins from various nyamiviruses and other mononegaviruses.

The third and fourth novel EVEs identified in our analysis encode predicted translation products similar to (−) ssRNA N proteins (Table 5). The predicted translation product of the first N-like EVE (Genbank accession number MF327148) is most similar to the N protein of a rhabdovirus isolated from the speckled wood butterfly (*Pararge aegeria*) [64]. This product is also similar to N proteins of several other insect and vertebrate rhabdoviruses. The product of the second N-like EVE (Genbank accession number MF327144) is most similar to the N protein of Taï virus, a mosquito bunyavirus [65], and is also similar to N proteins of several related insect bunyaviruses. Approximately 492 bps of the 699 bps Taï virus N-like ORF encodes a translation product that is similar to bunyaviral N proteins.

We identified homologous ORFs in several lepidopteran insects, suggesting this ORF may contain a conserved exapted viral gene. These homologous lepidopteran ORFs also contained a region that was recognized as a bunyavirus N-like by comparison to the NCBI CDD. Figure 7 shows the results of a phylogenetic analysis demonstrating the relationship among the product of the Sf ORF containing the Taï virus N-like EVE, related lepidopteran predicted proteins, and related bunyavirus N proteins. The lepidopteran gene products clustered closely together, whereas bunyaviral N proteins formed a distinct outgroup.

**Fig. 7:** Phylogenetic analysis of the Sf cell Taï virus N-like EVE product, homologous lepidopteran gene products, and related bunyavirus N proteins. The lepidopteran gene products cluster closely together in a group that is distant from the bunyavirus N proteins

The number of normalized reads mapped (RPKM) to the Sf Taï virus N-like EVE is much higher than the number mapped to other EVEs (Table 5). In fact, the RPKM value is more similar to the value observed with cellular genes, which supports the idea the Taï virus N-like EVE may be exapted. Lastly, whereas typical EVEs are not spliced, the mRNA encoding the Taï virus N-like EVE comprises three spliced exons (see Genbank accession number MF327150), further supporting the idea that the Taï virus N-like EVE is an exapted viral gene, or partially consists of an exapted viral gene.

Finally, the fifth novel EVE we discovered encodes a putative protein similar to the C-terminal half of the G protein of several bunyaviruses, most notably phleboviruses (Table 5). The predicted translation product of this G-like EVE (Genbank accession number MF327149) is most similar to the G protein of Shuangao Insect Virus 3 [66], and is also similar to G proteins from other bunyaviruses, including several other insect phleboviruses.

### Errantiviruses

Errantiviruses are not actually viruses, but a type of insect-specific long terminal repeat (LTR) retrotransposon. Errantiviruses are derived from typical LTR retrotransposons, which also contain *gag* and *pol* genes. However, errantiviruses have an additional third ORF encoding an env-like membrane fusion protein [67–74], which makes them similar to endogenous retroviruses in genome structure and organization. The *Drosophila* errantivirus *Gypsy* can form particles [75, 76], and it appears *Gypsy* can be transmitted horizontally to other individuals of the same and related species [76–81]. Thus, some errantiviruses can form particles and can potentially transfer genetic material to other cells under the right conditions.

FDA regulatory guidelines for the characterization and qualification of cell substrates specifically mention the quantity and type of retroviruses should be assessed [82, 83]. Considering the similarity between errantiviruses and endogenous retroviruses, insect cell substrates should also be screened for errantiviruses. This is underscored by the fact that several biologicals are produced using baculoviruses infection, which upregulates errantiviral transcripts [84–86].

Menzel and Rohrmann [18] previously identified several partial sequences similar to the reverse transcriptase domain of errantivirus POL proteins in Sf cells. However, the POL proteins of errantiviruses are very similar to those of typical LTR retrotransposons lacking a third env-like ORF. Thus, the partial sequences identified by Menzel and Rohrmann could be derived from either errantiviruses with a third env-like ORF, or from typical LTR retrotransposons lacking a third ORF. Menzel and Rohrmann also did not determine whether their partial sequences were associated with intact or partial, non-autonomous retrotransposons containing insertions, deletions, frameshifts, and/or nonsense mutations. Furthermore, because Menzel and Rohrmann PCR amplified these partial sequences from genomic DNA, it was not clear if they were actively transcribed.

The presence or absence of intact errantiviral sequences and their transcriptional status are important in determining their potential impact on the safety of biologicals produced in Sf-RVN cells. As errantiviruses are not classified as viruses, errantiviral proteins were not included in our VPD. To determine if Sf-RVN cells contain transcribed, intact errantiviruses, we used *Trichoplusia ni* TED [87] (a lepidopteran errantivirus) protein sequences and the previously identified partial Sf cell errantiviral sequences [18] as the query in a separate set of BLAST searches against the Sf-RVN cell genome and transcriptome.

We assembled a total of 13 distinct supercontigs containing all nine previously identified partial sequences, as well as some completely new sequences (See Additional file 1, Sf-Errantiviruses). Several of these supercontigs contained a (partial) third env-like ORF, indicating the previously identified sequences [18] were indeed derived from errantiviral, not typical LTR retrotransposons. Several of these env-like ORFs were intact and contained all the structural features required for functionality, i.e. a signal sequence, a C-terminal transmembrane domain, and a basic cleavage site. Several of the Sf-RVN errantivirus contigs comprised intact errantiviruses with LTR’s, a putative Ψ sequence, and intact *gag*, *pol* and *env* ORFs (ORFS 1–3) lacking any frameshifts or internal stop codons. Some contigs could not be completed, which might be due to either high similarity to other sequences or incomplete coverage. Some of these errantivirus sequences could also be partially identified in previously published Sf cell sequences [24, 25, 88]. We could not distinguish between highly similar sequences, therefore, it is possible that one or more of the sequences in our analysis are present in multiple copies or a number of highly similar variants.

A phylogenetic analysis based on an alignment of the predicted protein products of the Sf-RVN errantivirus sequences containing intact ORFs 1, 2 and 3 is shown in Fig. 8a. Figure 8b shows a phylogenetic tree for all identified errantivirus sequences, including those previously identified [18], based on an alignment of their DNA sequences. The relationships shown in these phylogenetic trees are similar to the previously reported relationships [18]. Notably, most Sf errantivirus sequences were closely related to TED, but two additional distinct clusters were identified. The first of these comprised Sf ErVs 2 and 12 (containing the previously identified Sf-70). The second additional cluster comprised Sf ErV 13, Sf-ErV 8 (containing Sf-20), and Sf ErV 5 (containing Sf-18). Thus, our data confirm and extend the previous conclusion that Sf cells contain diverse errantivirus families that are only distantly related to each other [18].

**Fig. 8:** Sf-RVN cells contain diverse transcribed errantivirus (ErV) sequences. **a** Phylogenetic analysis of Sf-RVN errantivirus sequences containing intact ORFs 1, 2 and 3 based on an alignment of the predicted protein products. **b** Normalized read abundances for Sf-RVN errantivirus sequences containing intact ORFs 1, 2, and 3. **c** Phylogenetic analysis of all identified Sf-RVN errantivirus sequences based on an alignment of their DNA sequences. Parentheses indicate previously identified sequences [20] found in the larger supercontigs assembled in this study (See Additional file 1, Sf-Errantiviruses)

All the distinct errantivirus sequences we identified were transcribed, albeit at different levels. Comparison of the normalized read abundances (reads per 1000 bps per million reads, RPKM) for errantiviral sequences containing non-interrupted ORFs 1, 2, and 3 showed there were nearly 100-fold differences in transcription levels (Fig. 8c). The level of transcription we observed for the distinct errantivirus sequences appears to correlate with the frequency at which Menzel and Rohrmann [18] isolated their partial sequences.

## Discussion

### Sf-RVN cells contain actively transcribed maverick transposons

We identified several transcribed virus-like sequences that are part of Maverick transposons, which are a novel class of giant transposable elements related to DNA viruses. Maverick elements are widespread in eukaryotes and have been identified previously in invertebrates including Lepidoptera [35]. The fact that Maverick transposons contain several ORFs encoding putative proteins very similar to proteins typically found in viruses has been previously noted and interpreted as evidence for ancient relationships between Maverick elements and various viral lineages [33, 89–91]. Our analysis of Sf Maverick elements extends these previously noted relationships with the observation that some insect Maverick elements encode a capsid-like protein (CAP) distinct from the previously described PY protein. We discovered CAP is related to parvoviral capsid proteins with an N-terminal PLA2 domain, including the *B. mori* densovirus capsid protein, which contains a jelly roll fold [92] that is also predicted to be present in the Maverick PY protein. We also uncovered an unexpectedly close similarity between *B. mori* densovirus DNA polymerases and insect Maverick DNA polymerases. Finally, we found entomopoxvirus capsid-like and ATPase proteins are similar to putative insect Maverick proteins. Taken together, our findings confirm and extend the previously identified close relationships between Maverick genes and various viral lineages.

### Transcribed retrotransposons could account for previously reported reverse transcriptase activity and might form particles

Reverse transcriptase (RT) activity was previously detected in Sf cells using highly sensitive PCR-based reverse transcriptase (PBRT) assays [93–95]. RT activity can indicate retrovirus contamination, but can alternatively indicate transcribed retrotransposons, which encode reverse transcriptase. For example, the POL protein encoded by the errantivirus TED ORF2 has reverse transcriptase activity [96]. The second ORFs of the related Sf-RVN cell errantivirus retroelements also contain RT domains, as determined by comparison to the CDD [22]. Thus, the errantivirus sequences we identified likely contribute to the RT activity detected in Sf cells. Moreover, TBLASTN searches with proteins from Baltimore Group VI and VII viruses identified many additional putative retroelements encoding proteins with RT domains, mostly Ty/Copia1 and Ty3/Gypsy family members. Retrotransposons are ubiquitous in both prokaryotic and eukaryotic genomes, and both retrotransposons and endogenous C-type retroviruses are endogenous to mammalian cell lines used to produce biologicals, such as CHO cells [97, 98]. Thus, Sf-RVN cells pose no greater biosafety risk than other cell lines that are use more commonly for biological manufacturing, such as CHO cells.

As the newly identified Sf-RVN errantivirus and Maverick sequences encode putative capsid genes that form particles, or could be encapsulated in virus-like particles (VLPs) [14], we suggest steps should be taken to ensure Sf cell-derived biologicals do not contain particles with intact errantivirus RNAs or Maverick DNAs. However, considering there is no evidence errantiviruses or Mavericks can form infectious particles that can productively infect mammals, including humans, the risk of horizontal errantivirus or Maverick transmission vectored through biologicals produced in insect cells is likely minimal or nonexistent.

### Comparison to other workflows

#### No reference cell genome is required

Workflows developed to probe for viruses in MPS datasets typically require a high quality reference cellular genome that is used to first subtract host cell reads from MPS datasets [4, 9, 10]. However, a ‘clean’, high quality reference genome is not always available. The use of parallel genome and transcriptome sequencing, as performed in this study, does not provide a reference genome for subtraction, as sequences from DNA viruses or proviral retroviruses would be eliminated in this filtering step and would therefore go undetected. As our workflow does not require a genomic subtraction step, it is suitable for species for which a high quality reference genome is not available. These include the insect cell lines used in the baculovirus insect cell system (BICS), such as Sf-RVN.

#### TBLASTN is more sensitive than BLASTN

Most workflows developed to probe for viruses in MPS datasets use the BLASTN algorithm as TBLAST searches are more computationally intensive and the results more difficult to interpret [6, 9]. However, the nucleotide sequences of unknown viruses might be only distantly related to viral sequences in the database, making their detection by BLASTN difficult, especially if only partial sequences of less conserved regions are represented.

In the present study, we discovered five novel EVEs. These are derived from viruses that have not been previously identified, or are extinct. Of these five novel EVEs, only one was similar to viral nucleotide sequences in GenBank, and could thus have been detected by BLASTN (Maraba virus L-like EVE, Table 5). The other four EVEs were not significantly similar to viral nucleotide sequences in GenBank, and could only have been detected by TBLASTN. Hence, the discovery of these four novel EVEs, which would not have been possible through BLASTN searches, underscores the utility of our method of using TBLASTN to detect sequences encoding viral-like proteins.

#### A minimum of 10 reads is required to detect virus-like sequences

Finding nucleotide sequences that encode predicted proteins similar to viral proteins by TBLASTN searching sequence assemblies has a sensitivity threshold determined by the minimal number of reads required to assemble contigs. We previously described four transcribed Sf-rhabdovirus-like endogenous viral elements (EVEs) in Sf9 and Sf-RVN cells [17]. The Sf-RVN cell genome assembled in this study contained contigs corresponding to these four EVEs. However, the Sf-RVN cell transcriptome assembled in this study only contained contigs corresponding to two of these four EVEs.

This apparent discrepancy can be explained by the low abundance of transcripts derived from these EVEs. Although only 2 transcribed contigs corresponding to Sf-rhabdovirus-like EVEs were assembled, read mapping showed that transcribed reads could be mapped to all four Sf-rhabdovirus EVEs. Specifically, 4, 14, 2, and 10 reads could be mapped to the N-, P-, G-, and L-like EVEs, respectively. The higher number of reads mapped to the P- and L-like EVEs (14 and 10) enabled the assembly of short contigs, whereas the lower number (4 and 2) mapped to the N- and G-like EVEs was insufficient for contig assembly. This demonstrates that as few as 10 reads can be sufficient to enable the detection of virus-like sequences in transcriptomic assemblies using our method.

The previously published transcriptome of Sf-rhabdovirus-contaminated Sf21 cells [25] was assembled from a total of 230 M reads, including 52,731 reads that could be mapped to the five Sf-rhabdovirus ORFs (11.9 kbps total). Considering our MPS data comprised 453.4 M reads, roughly 100,000 reads mapping to Sf-rhabdovirus ORFs could reasonably be expected if Sf-RVN cells were contaminated with this adventitious virus, and infection with another virus would probably result in a comparable number of reads. In context of the observation that our TBLASTN-based method has a sensitivity of ~10 reads, we suggest that if Sf-RVN cells were infected with one or more other viruses, there would have been sufficient viral sequence-specific reads for the assembly of contigs that would have been detected in our TBLASTN searches.

## Conclusions

### TBLASTN searching genome and transcriptome assemblies is sensitive and fast

Workflows developed to probe MPS datasets for viruses typically use very large sequence databases. These can comprise hundreds of thousands or even millions of sequences for use as queries in BLAST searches [4–6]. In contrast, our approach used a curated VPD of only a few thousand sequences specifically selected because they cover known viral diversity, with additional proteins from viruses known to infect insect cell cultures and *Spodoptera*. The use of this relatively compact dataset allowed us to manually cull sequences with cellular homologs. It also avoided the introduction of redundant sequences, or cellular sequences improperly annotated as viral. As a result, TBLASTN searches using the entire VPD against the complete WGS or TSA took only a few minutes on a typical PC. Furthermore, we were able to use an E value cut-off as high as 0.1. Thus, searching MPS assemblies for adventitious viruses with a compact, manually curated VPD is fast and yields sensitive results without requiring high performance hardware.

### No adventitious viruses were detected in Sf-RVN cells

While we detected various virus-like sequences in the genome and transcriptome of Sf-RVN cells, all were found to be components of Type I and II transposons, or were determined to be EVEs. We also were unable to detect any Sf-rhabdovirus sequences, which we readily detected in the published Sf21 cell transcriptome [25]. Furthermore, not a single read could be mapped to the Sf-rhabdovirus N, P, M, G, and L ORFs. Thus, our analysis confirms the previous conclusion that Sf-RVN cells are not contaminated with Sf-rhabdovirus or Sf-rhabdovirus variants.

Moreover, our analysis extends this conclusion by showing Sf-RVN cells are not detectably contaminated with any other adventitious viruses. The latter conclusion is strengthened by our discovery of novel short EVEs that are only distantly related to known viruses, which supports the notion that sequences derived from replicating viruses would have been detected, had they been present. The conclusion that Sf-RVN cells are not contaminated with any other adventitious viruses is further strengthened by the demonstration our approach is highly sensitive, requiring far fewer reads for a positive result than would be expected if Sf-RVN cells were in fact infected with a virus.

Thus, the overall results of this study strongly support the conclusion that Sf-RVN cells are a superior host for the production of safe biologicals for veterinary and human applications, as they harbor no Sf-rhabdovirus and most likely harbor no other adventitious viruses.

## Additional file

Additional file 1: The following supplementary files are part of this publication. (ZIP 77 kb)

## Abbreviations

BICS: Baculovirus insect cell system
CDD: Conserved domain database
EVE: Endogenous viral element
LINE: Long interspersed nuclear element
LTR: Long terminal repeat
MPS: Massively parallel sequencing
ORF: Open reading frame
PBRT: PCR-based reverse transcriptase
RPKM: Reads per 1000 bps of transcript per million mapped reads
RT: Reverse transcriptase
S1H: Superfamily 1 viral RNA Helicase domain
Sf: *Spodoptera frugiperda*
TSA: Transcriptome sequence assembly
VPD: Viral protein database
WGS: Whole genome shotgun
